# Circ‐SPECC1 modulates TGFβ2 and autophagy under oxidative stress by sponging miR‐33a to promote hepatocellular carcinoma tumorigenesis

**DOI:** 10.1002/cam4.3219

**Published:** 2020-07-06

**Authors:** Bin Zhang, Zhiyi Liu, Kuan Cao, Wengang Shan, Jin Liu, Quan Wen, Renhao Wang

**Affiliations:** ^1^ Institute of Digestive Diseases Xuzhou Medical University Xuzhou Jiangsu China; ^2^ Department of General Surgery Affiliated Hospital of Xuzhou Medical University Xuzhou Jiangsu China

**Keywords:** autophagy, circ‐SPECC1, HCC, miR‐33a, TGFβ2

## Abstract

Circular RNAs (circRNAs) play vital roles in the pathogenesis and development of multiple cancers, including hepatocellular carcinoma (HCC). Nevertheless, the regulatory mechanisms of circ‐SPECC1 in HCC remain poorly understood. In our study, we found that circ‐SPECC1 was apparently downregulated in H_2_O_2_‐treated HCC cells. Additionally, knockdown of circ‐SPECC1 inhibited cell proliferation and promoted cell apoptosis of HCC cells under H_2_O_2_ treatment. Moreover, circ‐SPECC1 inhibited miR‐33a expression by direct interaction, and miR‐33a inhibitor partially reversed the effect of circ‐SPECC1 knockdown on proliferation and apoptosis of H_2_O_2_‐treated HCC cells. Furthermore, TGFβ2 was demonstrated to be a target gene of miR‐33a and TGFβ2 overexpression rescued the phenotypes of HCC cells attenuated by miR‐33a mimics. Meanwhile, autophagy inhibition by 3‐methyladenine (3‐MA) abrogated the effect of miR‐33a mimics on proliferation and apoptosis of H_2_O_2_‐treated HCC cells. Finally, knockdown of circ‐SPECC1 hindered tumor growth in vivo. In conclusion, our study demonstrated that circ‐SPECC1 regulated TGFβ2 and autophagy to promote HCC tumorigenesis under oxidative stress via miR‐33a. These findings might provide potential treatment strategies for patients with HCC.

## Graphical abstract

We confirmed the specific role and molecular mechanism of circ‐SPECC1 in HCC and discovered that circ‐SPECC1 modulated TGFβ2 and autophagy under oxidative stress by sponging miR‐33a to promote HCC tumorigenesis.

## 1 INTRODUCTION

Hepatocellular carcinoma (HCC) is the major cause of cancer‐related death worldwide.^1^ Despite great advances in diagnosis and surgical treatment, the overall survival rate for HCC patients is still unsatisfactory due to its high recurrence rate.^2^, ^3^ Therefore, it is particularly urgent to develop novel therapeutics for the treatment of HCC.

Circular RNAs (circRNAs) are a class of noncoding transcripts with a covalently closed continuous loop.^4^ Accumulating evidence indicates that circRNAs are involved in the development and progression of human tumors.^5^ For example, hsa_circ_0008305 (circPTK2) was reported to hamper TGF‐β‐induced EMT process and metastasis via regulating TIF1γ in non‐small cell lung cancer (NSCLC).^6^ CircRNA ciRS‐7 facilitated the development and progression of esophageal squamous cell carcinoma (ESCC) by sponging miR‐876.^7^ Recently, hsa_circ_0000745(circ‐SPECC1), a novel discovered circRNA, was reported to promote tumorigenesis of gastric cancer cells via miR‐526b/KDM4A/YAP1 axis.^8^ However, the biological role of circ‐SPECC1 in HCC remains unknown.

Autophagy, a conserved catabolic process, is usually activated during adverse microenvironmental stress.^9^ During autophagy process, organelles with damaged structures and unwanted biomacromolecules are sent to lysosomes for digestion and degradation.^10^, ^11^ In addition, increasing evidence indicated that autophagy was closely associated with tumor development.^12^ For example, CLDN1 facilitated proliferation and migration of esophageal squamous carcinoma by inducing autophagy.^13^ MALAT1 facilitated colorectal cancer progression by activating autophagy.^14^ However, the regulation mechanisms about autophagy in HCC progression under oxidative stress are not fully understood.

In our study, we found that circ‐SPECC1 modulated TGFβ2 and autophagy under oxidative stress by sponging miR‐33a to promote HCC tumorigenesis. These findings will provide a novel theoretical basis for HCC treatment.

## 2 MATERIALS AND METHODS

### 2.1 Cell treatment

HepG2 and Huh‐7 cells were purchased from the Chinese Academy of Science Cell Bank (Shanghai, China). The cells were cultured in DMEM medium (Gibco), and supplemented with 10% of FBS in a humidified atmosphere containing 5% of CO_2_ at 37°C. To mimick the oxidative stress condition, 1 mmol/L of H_2_O_2_ was used to treat HCC cells for 12 hours. All experiments were approved by the Ethics Committee of the Affiliated Hospital of Xuzhou Medical University.

### 2.2 Cell transfection

The short hairpin RNAs (shRNAs) targeting circ‐SPECC1 (shcirc‐SPECC1) with control (shNC), miR‐33a mimics with control (miR‐NC), miR‐33a inhibitor with control (NC inhibitor), and pcDNA3.1/TGFβ2 with control (pcDNA3.1) were synthesized by Sangon. The transfection was performed using Lipofectamine 2000 (Invitrogen).

### 2.3 RT‐qPCR

Total RNA from HCC cells was extracted using TRIzol reagent (Invitrogen). For lncRNA and mRNA analysis, a Reverse Transcription Kit (Takara) was used to synthesize the first‐strand cDNA. For miRNA analysis, a miRNA First‐Strand cDNA Synthesis Kit (Sangon Biotech) was applied in the process of reverse transcription. The amplification reaction was operated in the SYBR‐Green PCR Master Mix kit (Applied Biosystems). The relative expression of genes was computed using the 2^−ΔΔCt^ method.

### 2.4 TUNEL

TUNEL Apoptosis Kit (Roche) was employed to assess cell apoptosis. After dehydrating by ethanol, HepG2 and Huh‐7 cells were dyed and cultured with TUNEL reaction mixture (Roche). The nuclear staining was performed with DAPI. A microscope (Olympus) was utilized to observe TUNEL‐positive cells.

### 2.5 CCK‐8

HepG2 and Huh‐7 cells were seeded into 96‐well plates with 5 × 10^5^ cells/well. Cell viability was detected at 0, 24, 48, and 72 hours. About 10 μL of CCK‐8 solution (Dojindo) was added into each well for another 4 hours. The absorbance at 450 nm was determined by a microplate reader.

### 2.6 Colony formation assay

Transfected HepG2 and Huh‐7 cells were added in 6‐well plates. After growing for 2 weeks, PBS (Sigma‐Aldrich) was used to rinse each well. Upon that, HCC cells were fixed in 4% of paraformaldehyde (Sigma‐Aldrich), and then, stained in 0.5% of crystal violet (Sigma‐Aldrich).

### 2.7 Western blot

Protein samples from cultured HepG2 and Huh‐7 cells were extracted using RIPA buffer (Beyotime) and separated by 10% of SDS‐PAGE. After transferring onto PVDF membranes, 5% of defatted milk was added. The membranes were incubated with primary antibodies against Beclin1 (ab210498; Abcam), p62 (ab56416, Abcam), and GAPDH (ab8245, Abcam) at 4°C overnight. Subsequently, membranes were incubated with secondary antibodies for 2 hours at room temperature. Protein bands were visualized using chemiluminescence detection system.

### 2.8 Luciferase reporter assay

The pmirGLO‐circ‐SPECC1‐Wt/Mut and pmirGLO‐TGFβ2‐Wt/Mut reporters were purchased from GenePharma. These reporters were cotransfected with miR‐33a mimics or miR‐NC into HepG2. After 48 hours, the activity of luciferase was evaluated by dual‐luciferase reporter assay system (Promega Corporation).

### 2.9 Autophagy inhibition by 3‐methyladenine (3‐MA)

HepG2 cells of miR‐33a mimics group were collected and subjected to incubation with DMEM complete medium containing 12.5 μg/mL of 3‐MA at 37°C and 5% of CO_2_.

### 2.10 Xenograft experiment

Male BALB/c nude mice (n = 6, 6 weeks old, ~20 g) were obtained from Shanghai SLAC Laboratory Animal Co., Ltd., and randomly divided into two groups. The HepG2 cells transfected with shNC or shcirc‐SPECC1 were injected subcutaneously into the flanks of each mouse. Moreover, xenograft tumor growth was detected and recorded every 7 days. The mice were sacrificed by cervical dislocation and tumors were collected for the following assays.

### 2.11 Statistical analysis

Data were presented as the mean ± standard deviation (SD). Each experiment was performed at least three times. Statistical analysis was carried out with SPSS 16.0 and GraphPad Prism. Comparisons between two groups were performed by a Student's *t* test. Comparisons among three groups were analyzed using one‐way ANOVA followed by Tukey's test. *P* < .05 was defined as statistically significant.

## 3 RESULTS

### 3.1 H_2_O_2_ inhibited circ‐SPECC1 expression and HCC tumorigenesis

To explore the effect of oxidative stress on HCC tumorigenesis, H_2_O_2_ was utilized to treat HepG2 and Huh‐7 cells. RT‐qPCR revealed that the circ‐SPECC1 expression was markedly decreased in H_2_O_2_‐treated HCC cells (Figure 1A). In addition, CCK‐8 and colony formation assays showed that H_2_O_2_ treatment suppressed the proliferation of HCC cells (Figure 1B,C). Moreover, TUNEL assays showed that H_2_O_2_ significantly promoted apoptosis of HCC cells (Figure 1D,E). To conclude, H_2_O_2_ downregulated circ‐SPECC1 expression and prevented HCC tumorigenesis.

**FIGURE 1:** H_2_O_2_ inhibited circ‐SPECC1 expression and HCC tumorigenesis. (A) Relative expression level of circ‐SPECC1 was examined by RT‐qPCR. (B and C) Cell proliferation was detected by CCK‐8 and colony formation assay. (D and E) Cell apoptosis was examined by TUNEL assay. ^*^ *P* < .05

### 3.2 Circ‐SPECC1 knockdown suppressed HCC progression under the treatment of H_2_O_2_

To investigate the specific function of circ‐SPECC1 in H_2_O_2_‐treated HCC cells, shcirc‐SPECC1 was transfected into HepG2 and Huh‐7 cells. RT‐qPCR showed that circ‐SPECC1 level was dramatically decreased in shcirc‐SPECC1 transfected HCC cells (Figure 2A). Subsequently, it was discovered that circ‐SPECC1 knockdown inhibited the proliferation of H_2_O_2_‐treated HCC cells (Figure 2B,C). TUNEL assay indicated that circ‐SPECC1 knockdown promoted apoptosis of HCC cells under H_2_O_2_ treatment (Figure 2D,E). These results indicated that circ‐SPECC1 contributed to tumorigenesis of HCC under oxidative stress.

**FIGURE 2:** Circ‐SPECC1 knockdown suppressed HCC progression under the treatment of H_2_O_2_. (A) The transfection efficiency of shcirc‐SPECC1 was evaluated by RT‐qPCR. (B and C) The proliferation of H_2_O_2_‐treated HCC cells transfected with shcirc‐SPECC1 or shNC was determined by CCK‐8 and colony formation assays. (D and E) The apoptosis rate of H_2_O_2_‐treated HCC cells transfected with shNC or shcirc‐SPECC1 was detected by TUNEL assay. ^*^ *P* < .05, ^**^ *P* < .01

### 3.3 Circ‐SPECC1 interacted with miR‐33a

To explore the molecular mechanism of circ‐SPECC1 in HCC, the downstream targets of circ‐SPECC1 were searched. With the assistance of starBase, the binding site of miR‐33a on circ‐SPECC1 was predicted (Figure 3A). Besides, overexpression of miR‐33a downregulated circ‐SPECC1 expression in HepG2 cells (Figure 3B). In addition, miR‐33a mimics obviously weakened the luciferase activity of wild‐type circ‐SPECC1, while had no influence on mutant circ‐SPECC1 (Figure 3C). Moreover, the miR‐33a expression was increased by H_2_O_2_ treatment in HepG2 and Huh‐7 cells (Figure 3D). To conclude, circ‐SPECC1 directly interacted with miR‐33a in HCC.

**FIGURE 3:** Circ‐SPECC1 interacted with miR‐33a. (A) The binding site between circ‐SPECC1 and miR‐33a was predicted by starBase. (B) The levels of circ‐SPECC1 and miR‐33a in HepG2 cells transfected miR‐NC or miR‐33a mimics were examined by RT‐qPCR. (C) Luciferase reporter assay was carried out to validate the combination between circ‐SPECC1 and miR‐33a in HepG2 cells. (D) The detection of miR‐33a level in H_2_O_2_‐induced HCC cells was performed by RT‐qPCR. *P < .05, **P < .01, ***P < .001

### 3.4 Silencing of miR‐33a partially restored shcirc‐SPECC1‐attenuated progression of HCC

To validate whether circ‐SPECC1 promoted HCC progression via miR‐33a, function assays were carried out. First, the upregulation of miR‐33a caused by circ‐SPECC1 knockdown was reversed by transfecting miR‐33a inhibitor into HCC cells (Figure 4A). Subsequently, it was found that miR‐33a inhibitor abrogated the inhibitory effect of shcirc‐SPECC1 on cell proliferation under oxidative stress (Figure 4B,C). Moreover, circ‐SPECC1 knockdown significantly enhanced cell apoptosis, which was abolished by miR‐33a depletion (Figure 4D,E). Overall, circ‐SPECC1 accelerated H_2_O_2_‐treated HCC cell progression by absorbing miR‐33a.

**FIGURE 4:** Silencing of miR‐33a partially restored shcirc‐SPECC1‐attenuated progression of HCC. (A) RT‐qPCR showed the relative miR‐33a expression of HCC cells transfected with shNC, shcirc‐SPECC1, and shcirc‐SPECC1 plus miR‐33a inhibitor. (B and C) CCK‐8 assay and colony formation assays were adopted to evaluate cell proliferation of H_2_O_2_‐treated HCC cells. (D and E) The cell apoptosis rate of H_2_O_2_‐treated HCC cells was assessed by TUNEL assay. ^*^ *P* < .05, ^**^ *P* < .01

### 3.5 TGFβ2 is a target of miR‐33a

The binding site between miR‐33a and TGFβ2 was predicted by TargetScan and was shown in Figure 5A. Additionally, luciferase reporter assay illustrated that the luciferase activity of cells with wild‐type 3’UTR of TGFβ2 was significantly reduced by miR‐33a overexpression while no alteration was observed in cells with mutant 3’UTR of TGFβ2 (Figure 5B). Besides, miR‐33a overexpression markedly decreased the mRNA level of TGFβ2 in HepG2 (Figure 5C). Moreover, the mRNA level of TGFβ2 was reduced in HepG2 cells by H_2_O_2_ treatment (Figure 5D). Overall, these results indicated that miR‐33a inhibited TGFβ2 expression through direct interaction.

**FIGURE 5:** TGFβ2 is a target of miR‐33a. (A) The binding site of miR‐33a on TGFβ2 3′UTR was presented. (B) The luciferase reporter assay was utilized to monitor the luciferase activity of wild‐type or mutant 3′UTR of TGFβ2 vector. (C) The level of TGFβ2 and miR‐33a in context of miR‐33a overexpression was examined by RT‐qPCR. (D) The TGFβ2 mRNA level in H_2_O_2_‐treated HCC cells was measured by RT‐qPCR. *P < .05, **P < .01, ***P < .001

### 3.6 MiR‐33a inhibited HCC progression by targeting TGFβ2

To confirm whether miR‐33a exerted its biological function by targeting TGFβ2, HepG2 cells were transfected with miR‐NC, miR‐33a mimics, and miR‐33a mimics + TGFβ2. According to RT‐qPCR, the downregulation of TGFβ2 induced by miR‐33a overexpression was abrogated by the overexpression of TGFβ2 in HepG2 cells (Figure 6A). In addition, the inhibitory effect of miR‐33a overexpression on cell proliferation was abolished by TGFβ2 overexpression under H_2_O_2_ treatment (Figure 6B,C). TUNEL assay revealed that TGFβ2 overexpression abrogated the promoting effect of miR‐33a mimics on HCC cell apoptosis in the presence of H_2_O_2_ (Figure 6D). In conclusion, our results demonstrated that miR‐33a modulated HCC cell proliferation and apoptosis by targeting TGFβ2.

**FIGURE 6:** MiR‐33a inhibited HCC progression by targeting TGFβ2. (A) RT‐qPCR showed the relative TGFβ2 expression in HepG2 cells transfected with miR‐NC, miR‐33a mimics, and miR‐33a mimics + TGFβ2. (B and C) CCK‐8 and colony formation assays were used to detected cell proliferation of transfected HepG2 cells under H_2_O_2_ treatment. (D) The apoptosis rate of H_2_O_2_‐treated HepG2 was analyzed by TUNEL assay. *P < .05

### 3.7 Autophagy inhibitor reversed HCC cell phenotypes induced by miR‐33a overexpression

We further investigated the regulatory mechanism of miR‐33a and autophagy in HCC. Western blotting results indicated that the transfection of miR‐33a mimics increased Beclin1 protein expression, but reduced p62 protein level, and miR‐33a depletion caused an opposite effect (Figure 7A). Moreover, 3‐MA (an autophagy inhibitor) partially abolished the inhibitory effect of miR‐33a mimics on cell proliferation (Figure 7B,C). By the same token, miR‐33a mimics‐mediated increased cell apoptosis was neutralized by 3‐MA (Figure 7D). In summary, autophagy inhibitor partially reversed miR‐33a overexpression‐induced cell proliferation inhibition and apoptosis promotion in HCC under H_2_O_2_ treatment.

**FIGURE 7:** MiR‐33a regulated the proliferation and apoptosis of HCC cells mediated by autophagy. (A) Western blot assay showed the protein levels of Beclin1 and p62. (B and C) Cell proliferation of H_2_O_2_‐treated HepG2 cells was evaluated by CCK‐8 and colony formation assays. (D) TUNEL assay was adopted to detect cell apoptosis of H_2_O_2_‐treated HepG2 cells. *P < .05

### 3.8 Circ‐SPECC1 knockdown prevented tumor growth in vivo

To determine whether circ‐SPECC1 could promote HCC progression in vivo, xenograft tumor experiment was performed. The results indicated that tumor size, weight, and volume were significantly reduced in shcirc‐SPECC1 group compared to shNC group (Figure 8A‐C). In addition, RT‐qPCR showed that depletion of circ‐SPECC1 downregulated the expression of circ‐SPECC1 and TGFβ2, whereas upregulated the expression of miR‐33a in tumors (Figure 8D‐F). In summary, circ‐SPECC1 promoted tumor growth in vivo.

**FIGURE 8:** Circ‐SPECC1 knockdown prevented tumor growth in vivo. The picture of tumors in vivo. (B and C) Tumor weight and volume was quantified. (D‐F) RT‐qPCR was carried out test the levels of circ‐SPECC1 miR‐33a, and TGFβ2 in tumors. *P < .05, **P < .01

## 4 DISCUSSION

With an increasing morbidity rate, HCC has led to approximately 600,000 death annually.^15^ Several factors, such as hepatitis B virus (HBV) and hepatitis C virus (HVC) infection, are related to the initiation of HCC,^16^, ^17^ but the pathogenesis of HCC remains unclear.^18^ Therefore, there is still a long way to explore the molecular regulatory mechanism in the tumorigenesis of HCC.

CircRNAs have attracted more and more attention and displayed their pivotal roles in various cancers, including HCC. For example, circ_0016788 was upregulated in HCC tissues and was associated with poor prognosis in HCC patients.^19^ Qiu et al indicated that circADAMTS13 acted as a molecular sponge of miR‐484 to suppress cell proliferation of HCC.^20^ Li et al found that circRNA MAT2B promoted HCC progression under hypoxic stress via miR‐338‐3p/PKM2 axis.^21^ Circ‐SPECC1 has been proved to act as an oncogene in a variety of cancers. Jiao et al indicated that circ‐SPECC1 facilitated the tumorigenesis of cervical cancer.^22^ Additionally, circ‐SPECC1 was upregulated in gastric cancer, which might function as a biomarker for gastric cancer treatment.^23^ In our study, we found that H_2_O_2_ downregulated circ‐SPECC1 expression and inhibited the HCC progression. Moreover, our research confirmed circ‐SPECC1 promoted cell proliferation but suppressed cell apoptosis of H_2_O_2_‐treated HCC cells, suggesting that circ‐SPECC1 acted as an oncogene in HCC under oxidative stress.

Increasing researches claimed that circRNAs could serve as a ceRNA to sponge miRNAs, thus regulating tumor development.^24^ For instance, Gao et al indicated that hsa_circRNA_0006528 accelerated breast cancer progression by sponging miR‐7‐5p.^25^ Meng et al reported that circSCAF11 accelerated the tumor growth via miR‐421/SP1/VEGFA axis in glioma.^26^ Similarly, we found that miR‐33a could bind with circ‐SPECC1 in HCC cells. Recent researches verified that miR‐33a inhibited breast cancer progression by regulating ADAM9 and ROS1.^27^ Additionally, miR‐33a suppressed the proliferation of NSCLC cells by targeting METTL3.^28^ Consistent with previous research, miR‐33a acted as a tumor suppressor in HCC by blocking the effect of circ‐SPECC1 on cell proliferation and apoptosis under oxidative stress.

TGFβ2 was a key effector in TGFβ/smad pathway,^29^ which has been reported to be implicated in the progression of HCC.^30^ For instance, Li et al reported that Bmi1 accelerated hepatocarcinogenesis by regulating TGFβ2/smad pathway.^31^ In our exploration, it was discovered that TGFβ2 was a target gene of miR‐33a, and TGFβ2 counteracted the impact of miR‐33a on proliferation and apoptosis in HCC cells under oxidative stress. Autophagy was proved to be closely associated with proliferation and apoptosis.^32^ However, the function of autophagy was controversial.^33^, ^34^ In our investigation, the addition of 3‐MA (an autophagy inhibitor) offset the tumor‐suppressive impact of miR‐33a on HCC, which indicated that autophagy could inhibit HCC development under oxidative stress. At last, animal assay demonstrated that circ‐SPECC1 knockdown prevented tumor growth in vivo.

In conclusion, we discovered that circ‐SPECC1 modulated TGFβ2 and autophagy under oxidative stress by sponging miR‐33a to promote HCC tumorigenesis (Figure 9). Nevertheless, this was just an initial exploration of circ‐SPECC1 in HCC, and further research of circ‐SPECC1 remained to be explored in future.

**FIGURE 9:** Schematic diagram shows regulatory mechanisms of circ‐SPECC1‐induced tumorigenesis of HCC

## CONFLICT OF INTERESTS

The authors declare that they have no conflict of interests.

## AUTHORS' CONTRIBUTIONS

Bin Zhang and Renhao Wang designed the study. Zhiyi Liu, Kuan Cao, and Wengang Shan performed the experiments. Zhiyi Liu, Jin Liu, and Quan Wen analyzed the data and prepared the figures. Bin Zhang and Renhao Wang drafted the manuscript. All authors approved this manuscript.

## Data Availability

The datasets used and/or analyzed during the present study are available from the corresponding author on reasonable request.
